# Role of fine-needle aspiration cytology in evaluating mediastinal masses

This article has been retracted.

**DOI:** 10.4103/0970-2113.56344

**Published:** 2009

**Authors:** D. K. Pandey, Zuber Ahmad, I. Masood, S. K. Singh, Z. Jairajpuri

**Affiliations:** *Department of TB and Chest Disease, J.N. Medical College, AMU, Aligarh, Uttar Pradesh, India*

**Keywords:** Fine-needle aspiration cytology, mediastinal mass, tissue diagnosis

## Abstract

**Background:**

Fine-needle aspiration cytology is an important and useful investigation and is considered next to imaging in the diagnosis of mediastinal lesions. We carried out this study in the Department of TB and respiratory diseases JNMC Aligarh from March 2000 to March 2002 with the following aims.

**Objectives:**

To make etiological diagnosis of mediastinal lesions, determine the pathological type of the tumor in cases of malignancy and evaluate the role of fine-needle aspiration cytology in staging of bronchogenic carcinoma.

**Materials and Methods:**

A total of 56 patients were included in this study who had mediastinal mass with or without lung lesions on chest X-ray or computed tomography scan. Of these patients, 36 had mediastinal mass only and 20 had mediastinal mass with parenchymal lesion.

**Results:**

In the present study, of 56 patients, 36 had mediastinal masses and 20 had pulmonary mass.

**Conclusion:**

Percutaneous fine-needle aspiration is an easy and reliable method for reaching a quick tissue diagnosis in pulmonary and mediastinal masses.

## INTRODUCTION

Fine-needle aspiration cytology (FNAC) was first used by Martin and Ellis[1] as a diagnostic tool. It is an important and valuable procedure for the diagnosis of lesion of thyroid, lymph node, bone, etc. FNAC has long been used for the confirmation of metastatic disease and in the diagnosis of primary mediastinal masses.

It can diagnose most lesions by accurate tumor typing. It has few complications and is relatively safe. It is particularly useful for the diagnosis of malignant lesions. The present study was undertaken to assess the role of FNAC in evaluating mediastinal masses. The aim and objective of the study were to cytologically characterize FNAC smears, to cell type the tumor in malignant cases, to correlate the findings and to aspirate mediastinal lymph nodes so as to stage the bronchogenic carcinoma.

## MATERIALS AND METHODS

The study was conducted in the department of TB and Respiratory disease, JNMC, Aligarh, from March 2000 to 2002. Fifty-six patients with mediastinal masses confirmed by computed tomography (CT) scan were included in this study. Of these patients, 36 had mediastinal mass only and 20 had lung lesion along with it.

FNAC was performed in each case. Percutaneous FNAC was performed in 20 patients, while CT-guided FNAC was performed in 36 patients. Percutaneous FNAC of mediastinal masses was conducted wherever mass was superficial enough to be approached percutaneously. For FNAC, a 22-gauge spinal needle with 20-ml sterile syringe was used. After fixation, slides were stained by one of the following methods, Hematoxylin and Eosin stain, PAP stain, Eosin Azure stain, Giemsa stain and specia stains such as Gram and Ziehl-Neelsen stain were used whenever necessary. Aspiration smears were studied for the probable diagnosis. Results of FNAC were correlated wherever possible with histological diagnosis.

## RESULTS

Maximum of number of cases were in the age group of 51-60 years with a mean age of 52 years. Male preponderance of 85.7% was seen. About 66.1% of total cases were malignant and 19.6% were benign [Table 1]. Benign lesions were inflammatory nonspecific (3.6%) and specific (5.2%). Two cases were diagnosed as specific inflammation, whereas actually there were three such cases. Among these three cases, two were diagnosed as granulomatous. Cytology revealed histiocytes of epitheloid type, forming cohesive clumps that were reminiscent of granuloma, with interspersed lymphocytes seen in one case. One case showed on cytology a cluttered background and necrosis. Numerous polymorphs were also seen. Fungal colonies with broad, folded non-septate hyphae were seen. A diagnosis of fungal abscess was favored.

**Table 1:** Distribution of cases according to nature of lesion

Nature of lesion	N	Percentage
Benign	11	19.6
Malignant	37	6.1
Unsatisfactory	8	14.3
Total	56	100

Retrosternal goiter was found in 3.6% cases, while ganglionuroma, mediastinal cyst, cystic teratoma, thymoma and reactive change lymph node comprised 1.8% each. Malignant lesions were cytologically characterized as carcinoma (50%), lymphoma (12.5%) and primitive neuroectodermal tumor (1.8%) [Table 2]. There were no false-positive cases because one case was falsely diagnosed as reactive change lymphadenopathy on cytology, thus giving a false-negative result. Later on, histopathological examination revealed the lesion to be non-Hodgkin lymphoma. FNAC of mediastinal masses was performed in all 56 cases, while histopathological examination was performed in 20 cases wherever required when the diagnosis was not clinically acceptable, hence ruling out the possibility of any false-positive cases. On cell typing, squamous cell was found to comprise 9 cases, adenocarcinoma 7, brochoalveolarcarcinoma 1, small cell carcinoma 10 and poorly differentiated carcinoma 1 [Table 3]. Small cell carcinoma was the most common type of carcinoma in our study. The correlation between cytology and histopathology was made in 20 cases, of which 19 cases were concordant and 1 was discordant [Table 4]. FNAC was inconclusive in 8 (14.3%) cases. Positivity of FNAC was 85.7%. Fortunately, no case of pneumothorax was encountered. This was confirmed in susceptible cases. While complications such as mild hemoptysis were encountered in 2 patients and chest pain in 14 cases.

**Table 2:** Distribution of cases according to the cytological diagnosis

Cytological diagnosis	N	Percentage
Benign lesions	12	21.4
Inflammation	5	-
Nonspecific	2	3.6
Specific	3	5.2
Mediastinal cyst	1	1.8
Retrosternal thyroid	2	3.6
Neurogenic tumor	1	1.8
Cystic teratoma	1	1.8
Thymoma	1	1.8
Reactive change	1	1.8
Malignant lesions	36	64.3
Carcinoma	28	50
Lymphoma	7	12.5
primitive neuroectodermal tumor	1	1.8
Unsatisfactory	8	14.3
Total	56	100

**Table 3:** Cytological types of malignant cases

Types	N	Percentage
Carcinoma	9	25
Squamous cell Ca	7	19.4
Adenocarcinoma	7	19.4
Bronchoalveolar Ca	1	2.8
Small cell Ca	8	22.2
Poorly differentiated	1	2.8
Combined carcinoma	2	5.6
Lymphoma		
Non-Hodgkin's lymphoma	5	13.8
Hodgkin's lymphoma	2	5.6
primitive neuroectodermal tumor	1	2.8
Total	36	100

Ca = Carinoma

**Table 4:** Cytological and histopathological correlation

Cytological diagnosis	N	Correlation	Concordant	Discordant
Benign lesions	12			
Inflammation	5	-	-	-
Nonspecific	2	-	-	-
Specific	3	1	1	-
Mediastinal cyst	1	-	-	-
Retrosternal thyroid	2	2	2	-
Neurogenic tumor	1	1	1	
Cystic teratoma	1	1	1	-
Thymoma	1	1	1	-
Reactive change	1	1	-	1
Malignant lesions	36			-
Carcinoma	28	5	5	-
Lymphoma	7	7	7	-
PNET	1	1	1	-
Unsatisfactory	8	-	-	-
Total	56	20	19	1

PNET = Primitive neuroectodermal tumor

## DISCUSSION

In our study, 56 FNAC from different compartments of the mediastinum were evaluated over a 2-year period. Of these cases, 19.6% were benign and 66.1% were malignant.

The study showed that the maximum number of cases was seen in the age group of 51-60 years. The increased number of cases in the age group of 51-60 years may be due to increased incidence of malignancies in that group and also because FNAC was mainly used for the diagnosis of neoplasm, which comprises 66.1% of the total cases. The average age in our study was 52 years. Powers *et al.*,[2] in their study also showed increased prevalence of neoplasm after age 50 years, with average age of 54 years; 71% of total cases were found to be malignant.

Maxcy Rosenau's last[3] study indicated that an experimental increase in the incidence rates with age is observed for most adult malignancies. This is true as increased number of malignant cases is seen in the elderly population.

Our study also showed that mediastinum is the site for a variety of lesions, both benign and malignant. Of 56 cases, 11 (19.6%) were benign and 37 (66.1%) were malignant, while 8 cases (14.3%) were inadequate for reporting. The malignant cases formed the largest category, and in this category metastasis was found in 50% of cases. A study conducted by Blegard *et al.*[4] also showed an appreciable proportion of malignant mediastinal tumors (30%). Similar results were also shown by Adler *et al.*[5] and Jareb *et al.*,[6] who reported a 72% prevalence of malignant disease in their study, which is comparable to 66.1% of the present study [Table 5].

**Table 5:** Prevalence of malignant tumor in mediastinal biopsies

Cell type	Authors		
	
	Lange *et al*. (1972) %[7]	Bocking *et al*. (1995) %[8]	Present study%
Squamous cell carcinoma	91	86.6	89
Adenocarcinoma	100	89.5	85.7
Small cell carcinoma	86	94.2	100

As is evident from the above table, squamous cell carcinoma, adenocarcinoma and small cell carcinoma can be effectively typed by cytology. A high degree of accuracy in cytological typing can be of great importance in those cases where no confirming histology is available. The highest typing accuracy was seen with small cell carcinoma and may be attributed to abundant material and characteristic cytological appearance. The carcinomatous lesions represent metastatic disease from thoracic and extrathoracic sites. Maximum cases originated from a lung primary (82%), while larynx, esophagus, stomach, colorectal and cervical primary represented 3.6% cases each. Thirty cases (maximum) were confirmed to the anterior compartment, 16 cases to the middle and 2 cases to the posterior compartment. Percutaneous FNAC, transbronchial needle aspiration (TBNA) and CT-guided FNAC were used to obtain material for cytology. Best results were obtained with CT-guided FNAC with just 1 inadequate yield, while TBNA had 2 and percutaneous FNAC showed a maximum of 5 inadequate samples.

One of the most important factors in the treatment of bronchogenic carcinoma is its curative resection. Because the tumor must be confined to the lung to be resectable and as the initial route of spread of most bronchogenic tumors is to mediastinal lymph nodes, thorough examination of the mediastinum is central to the assessment of resectability. FNAC of mediastinal lymph nodes is a reliable alternative to more invasive surgical staging techniques to prove the presence of mediastinal metastasis. The presence of lymphocytes in the aspirate was considered an essential criterion of specimen adequacy. Five cases of lymph node aspirate with lymphocytes in the background were obtained in our study and all were positive for malignancy, indicating unresectability and no further surgical procedure was undertaken. This highlights the role of FNAC in staging of bronchogenic carcinoma.

Complications of all 3 types of procedures were minor, such as pain and hemoptysis.

Verification of cytological diagnosis was made by histopathological examination wherever possible and therapeutic response to relevant therapy in the remaining cases.

The study concluded that FNAC of mediastinal masses is a relatively safe and easily tolerated procedure, particularly for the diagnosis of mediastinal tumors such as malignant lesions. CT-guided FNAC is the most successful procedure, whereas TBNA is very effective in staging bronchogenic carcinoma. In view of the above study, it is recommended that FNAC should be the first invasive procedure for the patients of mediastinal masses.
